This article has been retracted.

# A Signature of Genes Featuring *FGF11* Revealed Aberrant Fibroblast Activation and Immune Infiltration Properties in Keloid Tissue

**DOI:** 10.1155/2022/4452687

**Published:** 2022-08-09

**Authors:** Bo Yuan, Linlin Miao, Disen Mei, Lingzhi Li, Zhu Hu

**Affiliations:** ^1^Dermatology Department, The Affiliated Hospital of Medical School, Ningbo University, No.247 Renmin Road, Jiangbei District, Ningbo 315020, China; ^2^Surgery Department, School of Medicine, Ningbo University, No.818, Fenghua Road, Jiangbei District, Ningbo 315211, China; ^3^Basic Medicine Experiment Center, School of Medicine, Ningbo University, No.818, Fenghua Road, Jiangbei District, Ningbo 315211, China; ^4^Plastic and Reconstructive Surgery Department, The Affiliated Hospital of Medical School, Ningbo University, No.247 Renmin Road, Jiangbei District, Ningbo 315020, China

## Abstract

Keloid is a fibroproliferative disorder in the skin, which manifested with extensive deposition of collagen and extracellular matrix. Its etiology remains a mystery and its recurrence rate remains high despite combinative treatment regimens. Current hypotheses of its pathogenesis centered on the role of inflammatory processes as well as immune infiltration in the microenvironment. However, there are a lot of discrepancies when it comes to the verification of certain well-recognized pathways involved in the dysfunctional fibroblast. Further exploration and characterization are required to reveal the driving force and even leading genes responsible for keloid formation. In this study, we provided supportive evidence of the immunologic nature of keloids distinct from normal fibroblasts and physiological scars by incorporating multiple available expressional profiles in the Gene Expression Omnibus (GEO). Through differential analyses and functional analyses, we identified a set of genes that successfully captures the dissimilarities between keloid lesions and nonlesions. They were differentially regulated in keloid samples and had opposite behavior in exposure to hydrocortisone. A key signature of six genes featuring *FGF11* not only was highly correlated with significantly dysregulated fibroblast activation but also reflected various levels of immune cell infiltration. *FGF11*, in particular, revealed the heterogenous immunologic nature of keloid lesions. This study further supported that aberrant fibroblast was one of the main contributing factors and shed some light on investigating immune properties in future studies.

## 1. Introduction

Damaged tissue undergoes a complicated process of repair and regeneration till the wound is healed, which starts right after the skin injury and can consume a significant amount of time. Under pathological circumstances like excessive collagen deposition, hypertrophic scars or keloids develop. The exact mechanism of abnormal wound healing processes has yet to be clarified. In most cases, the differences between keloid and hypertrophic scars can be understood by clinical observation, in that hypertrophic scars remain within the confines of the original wound. In contrast, the keloid extends way beyond the boundaries of the injury [1]. However, there are more distinctive features of keloid underlying a significantly different nature of it than hypertrophic scars. The keloid pathology is not well understood but has been speculated to be related to the imbalance between collagen synthesis and degradation [2]. The most common vulnerable sites to keloid include the earlobes, presternal skin, and all areas with no hair follicles or other glands. A wide range of types of skin injuries seem to be responsible, but no particular type has been specified to be associated with keloid formation. Keloidogenesis can arise even without any antecedent injuries [3]. Researchers suspect that consistent inflammation near the injured site can induce fibroblast malfunction, hindering the scar's maturation. The inability of the fibroblast within keloid tissue to respond normally to stimulation triggers the resistance of the keloid to treatments and high rates of recurrence [4].

Keloids, most of the time, occur as sporadic cases but can be familial [5]. Its high occurrence in darker-skinned ethnicities suggests a genetic predisposition or even a hereditary component in the pathogenesis. Both autosomal recessive and dominant modes have been proposed, but these studies' scale is too narrow to draw convincing conclusions [6, 7]. Moreover, single nucleotide polymorphisms and other epigenetic mechanisms have also been associated with keloidogenesis [8].

Most hypotheses about the formation of keloids focus on the overproduction and excessive deposition of collagen. Still, an increasing body of evidence shows the importance of the inflammatory and immunologic responses as potential initiators of this pathologic process. High concentrations of infiltrating inflammatory cells [9] and comorbidities with autoimmune disorders [10] indicate the value of exploring the correlation between dysregulated inflammatory responses and aberrant immune function execution.

Although keloid is labeled as an abnormal but benign dermal growth where excessive scar tissue results from failed suppression of wound healing, it resembles malignant tumor cells in terms of its hyperproliferative nature and capability of invasion. There is also growing evidence showing that keloid-prone populations, especially males, face a significantly higher risk of developing skin malignancies [11]. This, along with the cosmetic burden and disabling potential of large keloids, entails more advanced, effective treatment regimens. However, despite the efforts that have been put into the research of the pathophysiology of keloid formation, it is still unclear what modulators or pathways are controlling the process. The mainstay of currently available therapies is to reduce the keloid recurrence, but the optimal results cannot be achieved unless its mechanism gets unrevealed.

Therefore, in this study, we incorporated multiple available expression profiles associated with keloids and conducted a series of bioinformatical analyses to further explore the immune properties of keloid lesions. A small signature of genes featuring *FGF11* was found to be differentially regulated in keloids with a different pattern under hydrocortisone treatment and depicted the increased lymphocyte infiltration in keloid lesions. Furthermore, the expression level of *FGF11* also reflected the heterogenous nature of keloid lesions in terms of immunologic signatures. This study reinforced the importance of investigating the role of Th1 and Th2 balance and brought up the necessity of observing keloid development dynamically. The shortage of the latter could have contributed to some current discrepancies on this inflammatory fibroproliferative disease.

## 2. Materials and Methods

### 2.1. Datasets

One expression profile acquired from Gene Expression Omnibus (GEO) was adopted (GSE7890, available at https://www.ncbi.nlm.nih.gov/geo). Samples in this dataset included keloid fibroblasts and normal scar tissue, with or without hydrocortisone treatment. To validate the value of identified differentially expressed genes (DEGs) in identifying the differences between keloid and nonkeloid lesions, GSE92566 was accessed from the same database. The expression matrix of six samples containing three biopsies of large keloid lesions and their adjacent nonlesioned skin samples from GSE92566 was used. The batch effect was removed and these two expression profiles were merged into a larger dataset to further explore the functional pathways implied by the aberrant expressions of these genes. GSE121618 was also used to investigate the microenvironment of epithelial samples from keloid patients versus healthy control.

### 2.2. Differential Analyses

We separated the expression matrix available from GSE7890 into two groups and compared them based on limma analysis [12]. Group 1 was keloid samples without hydrocortisone treatment versus normal scar tissue with no treatment; Group 2 was between treated and untreated keloid samples. The absolute fold change value (FC) was set as 2, shown as |Log2FC| > 1 in figures, and a *p* value less than 0.05 was considered statistically significant.

### 2.3. Gene Ontology Analyses

Gene ontology (GO) enrichment analysis was conducted on the DEGs in R (version 3.1.0). GO annotation was acquired through the R package “org.Hs.eg.db” and the actual enrichment process was analyzed with package “clusterProfiler” (version 3.14.3). Major molecular functions of DEGs were presented, and *p* value = 0.05 was set as the threshold.

### 2.4. Immune Infiltration Score

One algorithm named xCELL [13] was applied in this study to calculate the infiltration scores of different types of cells (primarily immune cells and stromal cells) and immune scores and microenvironment scores.

### 2.5. Gene Set Variation Analysis

To reveal the alterations of major pathways involved in fibroblast functions, four sets of functionally curated genes were acquired from the Molecular Signatures Database (https://www.gsea-msigdb.org/gsea/msigdb/index.jsp). These included gene sets: GOBP_FIBROBLAST_ACTIVATION, GOBP_FIBROBLAST_PROLIFERATION, GOBP_FIBROBLAST_APOPTOTIC PROCESS, and GOBP_FIBROBLAST_MIGRATION. Genes involved in these processes were considered a signature profile. Based on these signatures, gene set variation analysis (GSVA) was performed, and enrichment scores were calculated.

### 2.6. Gene Set Enrichment Analysis

Differential analyses were first conducted to acquire the fold changes in gene expression (1) between keloid lesions and nonlesion keloids; and (2) between keloid samples expressing high or low level of *FGF11* (separated by 50% median). Then, GSEA analyses were conducted based on annotations from Hallmark gene sets and c7 (immunologic signatures) from the molecular signatures database (MSigDB, v7.2).

### 2.7. Correlation Analyses

Pearson's correlation analyses were performed to explore the following relationships: (i) expression levels of key genes and biological processes associated with fibroblast function; and (ii) expression levels of key genes and infiltration scores of immune-related cells calculated by xCELL.

### 2.8. Cell Lines

KEL FIB (CTCC-001-0209) and BJ (CTCC-400-0144) cells were purchased from MeisenCTCC (Zhejiang, China). KEL FIB cells are keloid fibroblasts acquired from a 35-year-old black women, while BJ cells are fibroblasts established from the normal foreskin of a male neonatal. Keloid fibroblasts were cultured in Dulbecco's modified Eagle medium (DMEM) containing 10% fetal bovine serum (FBS), 100 U/ml penicillin, and 100 *μ*g/ml streptomycin in a humidified incubator with 5% CO_2_ and 95% air at 37°C.

### 2.9. Quantitative Polymerase Chain Reaction (qPCR)

Total RNAs were extracted from cell cultures, and cDNAs were subsequently synthesized with HiScript II First Strand cDNA Synthesis Kit from Vazyme Biotech Co., Ltd (Nanjing, China), following the manufacturer's instructions. The qPCR was performed using Taq Pro Universal SYBR qPCR Master Mix Kit from Vazyme Biotech Co., Ltd (Nanjing, China), matrix and the following primers were used: H-IGFBP5-F4 (5′-CAAGAGAAAGCAGTGCAAACC-3′), H-IGFBP5-R4 (5′-AGGTGTGGCACTGAAAGTCC-3′); H-FGF11-F4 (5′-CCTCAGCTCAAAGGCATCGT-3′), and H-FGF11-R4 (5′-CAGGTTGAAGTGGGTGAAGGA-3′). Actin *β* was chosen as the internal reference and the following primers were used: H-ACTB-F2 (5′-CTCCTTAATGTCACGCACGAT-3′) and H-ACTB-R2 (5′-CATGTACGTTGCTATCCAGGC-3′). Experiments were designed and repeated with three biological replicates, each of them containing three technological replicates.

### 2.10. Statistical Analyses

For comparisons among multiple groups, one-way analysis of variance (ANOVA) or Kruskal–Wallis one-way ANOVA was used when applicable. Dunn's multiple-comparison corrections were adopted for post hoc comparisons. For comparisons between two groups, Student's *t-*test or Mann–Whitney test was used when applicable. A *p*value less than 0.05 was considered statistically significant in all situations.

## 3. Results

### 3.1. Identification of Genes Differentially Upregulated in Keloid Tissue but Downregulated in Treated Keloids

The volcano plots in Figure 1 show significantly (|Log2FC| > 1, *p* < 0.05) up or downregulated genes during comparisons between (1) keloid samples without hydrocortisone treatment and normal scar tissue without treatment (Figure 1(a)) and (2) treated and untreated keloid samples (Figure 1(b)). Totally 167 genes were significantly downregulated under the influence of hydrocortisone treatment compared with keloids without exposure to it. What is more, of the 112 genes upregulated in keloid tissues compared with normal scar, 22 were significantly downregulated after hydrocortisone treatment (Figure 1(c)). Some of these genes were functionally enriched to insulin-like growth factor (IGF)-binding and other growth factor-binding pathways (Figure 1(d), Table 1).

We verified the actual expression levels of these 22 DEGs in the abovementioned four conditions. As shown in Figure 2(a), except for *KCND3* (*p*=0.07), *LRRC17* (*p*=0.35), and *RHOJ* (*p*=0.10), the rest of these genes were expressed at statistically different levels. Specifically, for the comparisons within groups, *CA12* (*p*=0.02), *CAMK1D* (*p*=0.01), *ESM1* (*p*=2.7*e* − 3\), *FGF11* (*p*=0.03), *FOXP1* (*p*=0.04), *GXYLT2* (*p*=0.03), *HOMER1* (*p*=0.04), *IGFBP5* (*p*=0.03), *KIT* (*p*=0.04), *MEST* (*p*=0.04), and *RAB3B* (*p*=0.04) were consistently expressed at statistically different levels between keloids without hydrocortisone and normal scar tissue without treatment. In paired keloid lesion samples given hydrocortisone treatment, most of them were comparatively lower than the statistically significant level except *HOMER1* (*p*=0.06*p* *=* 0.06), *KIT* (*p*=0.05), *MEST* (*p*=0.05), and *RAB3B* (*p*=0.05).

The dimensionality of the expression profile consisting of 22 DEGs was reduced and depicted with principal component analyses (PCA) at the two-dimensional and three-dimensional levels (Figures 2(b) and 2(c), respectively). The distinct features of keloid lesions and nonlesions could be observed well from the separated clusters in both levels. Collectively, these results indicated that these DEGs represented a possible trend existing in keloids different from nonlesions.

### 3.2. Keloid Lesions Exhibited Patterns of Aberrant Activation of Fibroblast and Increased Immune Infiltration

We next investigated if the following signatures involved in fibroblasts were aberrantly changed in keloids: proliferation, activation, migration, and apoptosis. Compared with physiologic scars, keloid samples (regardless of the lesioned situation) exhibited significantly increased activation of fibroblast (*p*=0.05, Figure 3). There was no significant up- or downregulation of the rest of the three signatures. With a threshold of *p* less than 0.01 and a correlation coefficient over 0.60, *ARHGAP29*, *C4orf47*, *DOK3*, *FGF11*, *MEST,* and *PFKFB4* were significantly correlated with the activation of fibroblast positively (Figure 3) Because the expression levels of these genes are also elevated in keloids compared with normal scars, these genes may contribute to the proliferative phase in the early formation of keloids by promoting fibroblast activation.

We further explored the cells infiltrating the microenvironment of keloids. The algorithm named xCELL was used to calculate a wide range of scores from the overall immune scores to individual infiltration scores of different cells. A merged cohort including GSE7890 and GSE92566 plus another one focusing specifically on epithelial cells were used at this stage. The key genes identified above were also significantly correlated with infiltrating scores of lymphocytes and major proinflammatory cells (Figure 4). With a threshold of *p* less than 0.05 and a correlation coefficient over 0.60, CD4^+^ naïve T cells, CD4^+^ Tcm cells, CD4^+^ Tem cells, CD8^+^ T cells, class-switched memory B cells, DC, mast cells, iDC, pro-B cells, and the overall Th1 cells and Th2 cells were included. *FGF11* consistently correlated with the infiltration scores of CD4^+^ Tcm cells, iDC, pro-B cells, and the overall Th2 cells when the subject of expressional profiling was purified epithelial cells. The previously weak negative correlations between *FGF11* and fibroblast, macrophages, and pDC became additionally significant. While most of the correlations were in a similar fashion as they were in mixed keloid lesions and nonlesions, some became the opposite in GSE121618. The most noticeable ones would be the correlations between gene *DOK3* and CD4^+^Tcm cells, CD8^+^ T cells, and neutrophils. Interestingly, the overall immune score of keloid lesions was significantly higher than that of nonlesion samples (*p*=0.01), but the opposite was observed between keloid epithelial samples versus normal epithelial cells.

We wanted to further capture the functional differences between keloids and nonlesions. From the merged cohort containing both keloid and its nonlesion control, significantly enriched well-defined biological states or processes from Hallmark and curated immunologic signature gene sets from C7 were identified. Representative gene sets and processes are shown in Figure 5. Significantly different enrichment of processes associated with mitotic cell spindle, G2M checkpoint, and apoptosis was observed (not shown). On the other hand, up to 163 immune-related gene signatures were also enriched according to c7 curated sets; they were mainly centered on the function of proinflammatory cytokines and lymphocytes such as Th1, Th2, and Th17 cells.

### 3.3. Potential Role of FGF11 in Driving the Altered Immune Properties in Keloids

In the previous correlation analyses, *FGF11* is consistently correlated with major lymphocyte lineages. Of all identified key genes, it is also the only one in the complete list of immune-related genes curated by ImmPort (updated in July 2020, ID 2256, available at https://www.immport.org/shared/genelists). Thus, we again explored the possible differences in gene enrichment between keloid samples with higher FGF11 and those with lower levels (Figure 6). Consistently significant differences in hallmark processes related to the mitosis and proliferation of cells were observed. Responses to interferon-alpha and gamma were also significantly enriched (ES = −0.515, *p*=0.007; ES = −0.469, *p*=0.007, respectively) in addition to hypoxia-related processes (ES = 0.493, *p*=0.005) and inflammatory responses (ES = −0.464, *p*=0.007). We also verified its expression between keloid-derived fibroblasts and normal fibroblasts with PCR (Figure 7). The expression level of FGF11 in our experiment was significantly lower in keloid fibroblasts (*p*=0.0171), which was consistent with what was observed in keloid epithelial cells overall, contrary to the trend observed in keloid tissue (Figure 7). Another gene, *IGFBP5,* that was possibly associated with the proliferative stage of keloid development, identified in our first step, was also tested. Even though the IGF pathway has been long suspected to be important in keloidogenesis, the role of IGFBP5 has been inconsistently reported. In our PCR analysis, it was significantly lower in keloid fibroblasts (*p*=0.0006), opposite to the trends universally observed in the rest of the expression profiles.

## 4. Discussion

An abnormal wound healing process can induce the development of keloid, a fibrous hyperplastic skin disease. While keloid exhibits similar histological features as hypertrophic scars, it behaves like malignant tumors with the ability to invade deeply and extend beyond the wounds' original edge. The pathophysiology of keloid development is still under investigation, but it is speculated to be rather complex. Overall, excessive collagen deposition could be observed as a primary characteristic manifestation. Health concerns from keloids have been mostly centered on cosmetic defects and intense itching or pain in some patients. It has a high prevalence of recurrence despite various treatments available clinically. Keloids grown in certain areas can also become symptomatic by limiting joint mobility and even causing deformity. Although keloids have been considered benign, growing evidence shows that the underlying pathogenesis and recurrent episodes entail regular skin examinations as the keloid-prone population faces a significantly higher risk of developing skin cancer, especially males [11].

Fibroblast has been presumed to be the primary cell driving this abnormal excessive collagen formation [9]. After all, it is a significant component of keloid tissues with a significantly higher concentration than normal tissues [14]. Fibroblasts are usually recruited near the wound or differentiated from resident stem cells in the very early stages of wound healing. Imbalanced proliferation and apoptosis of keloid fibroblasts might have contributed to the increase in cell content, hypersecretion of cytokines from keloid fibroblasts, and high sensitivity of themselves to other signal transductions also play an important role [15–17]. Zhang et al. have revealed higher levels of proliferation of keloids compared with physiological scars and normal tissue, but the apoptosis levels seemed to be similar [18]. However, this observation might be opposite in different stages or regions of keloids as there is other evidence showing decreased apoptosis plus higher proliferation in early keloids [19]. This indicates that the relationship between apoptosis and proliferation of keloid fibroblasts could be dynamic, and a reversed pattern of high apoptosis in addition to low proliferation might prevent keloids from becoming malignant. The balance can also be reachieved when treatments such as hydrocortisone are introduced into the microenvironment of keloids. In our study, we specifically focused on the part of the gene profile that was upregulated in keloid scars compared with normal scars, which was also downregulated under hydrocortisone; they depicted the key molecular functions such as IGF binding, integrin binding, ion channel binding, and other growth factor binding. From the work of Zhang et al. mentioned above, we did not find significant differences among keloid lesion, nonlesion, and physiological scar in terms of the apoptotic profile of fibroblast. Meanwhile, fibroblast activation, instead of aberrant proliferation, was revealed to be significantly higher in keloid-prone subjects. This was highly correlated with the expression levels of DEGs identified between keloid and nonkeloid that were also potentially regulated under the influence of hydrocortisone.

IGF pathway is crucial for cell proliferation and growth. Some IGF-binding proteins (IGFBPs) and IGF receptors have been hypothesized to be therapeutical for malignancies. IGFBP-2 through 5 have been frequently associated with the pathogenesis of keloids, but their exact functional significance in the skin has not been clarified [20–22]. The influences on the activities of IGF can be either inhibitory or enhancing, which will lead to either anti or proapoptotic effects on fibroblasts. We verified the expression level of *IGFBP5*, one major gene within the group of DEGs associated with the IGF pathway. In commercially available keloid fibroblasts, its expression turned out to be significantly higher than that of BJ cells, normal fibroblasts derived from the normal foreskin. This supports the negative correlation previously identified between *IGFBP5* expression and fibroblast proliferation induced by keloid keratinocytes [23].

As an inflammatory fibroproliferative process, keloid formation is believed to be under regulation by a series of inflammatory cytokines released by proinflammatory cells or immune cells infiltrated in the microenvironment of keloids or lesions with a potential to become keloids. Macrophages play a crucial role in the wound healing process, and the adjustment of inflammation versus tissue repair partially relies on the balance between M1 and M2 [24, 25]. High infiltration of macrophages and lymphocytes was observed in keloid specimens, and M2 was consistently the dominant type [26, 27]. Using the xCELL algorithm, we explored the infiltration of major cell types of lymphoid and myeloid lineages in the microenvironment of both keloid lesions and nonlesion keloids. Samples collected from keloid lesions had significantly higher immune scores than those collected from nonlesion areas. Most of the DEGs significantly correlated with the activation process of fibroblast (*p* < 0.01, correlation coefficient over 0.6) were highly correlated with the infiltration of CD4-positive naïve T cells, central memory T cells (Tcm), effector memory T cells (Tem), CD8-positive T cells, dendritic cells, and mast cells. They also exhibited significantly opposite correlations with Th1 and Th2 cells. In terms of the balance of M1 and M2, though not significantly correlated, these genes seem to affect the two types of macrophages in opposite directions. However, the immune landscape was reversed when we repeated similar scoring and correlation analyses in GSE121618, where epithelial cell samples acquired from keloid patients and healthy subjects were employed. The opposite effects of the key DEGs on Th1 and Th2 cells also failed to be observed. Currently available studies have agreed on the promotive effects of Th2 cytokines such as interleukin 4 and interleukin 13 on the development of fibrosis [28]. However, whether they control the direction of keloid progression extensively is debatable. Their low expression profiles in both keloid and normal fibroblast, and the clinical evidence of the failure of medications that specifically block Th2 cytokines [29, 30], all necessitate further explorations in the balance of Th1 and Th2 responses. Again, consistent with a hypothesis mentioned earlier, a cross-sectional observation of these samples might be inadequate if keloid development is a dynamic process in terms of the balance between Th1 and Th2. The inconsistent actual expression levels of key genes such as *FGF11* might be associated with the stages of keloid samples.

With that being said, the aberrant nature of immune responses within keloids could be appreciated from our GSEA analyses. What is more, *FGF11* consistently correlated with Th2 cell infiltration in mixed tissue samples or epithelial cells; thus, it was selected as the grouping factor to conduct single-gene GSEA. Interestingly, this gene depicted the heterogenous immune properties of keloids, even though the function of this gene, especially in the skin, is yet to be determined. As a member of the FGF family, it possesses broad mitogenic and cell survival activities, including cell growth, morphogenesis, tissue repair, tumor growth, and invasion, and is reasonable to hypothesize the role of *FGF11* in regulating tissue repair and fibrosis in keloidogenesis [31]. However, despite repeated validation of the PCR results for FGF11 in this study and the selection of more appropriate primers, the peak pattern of the lysis curve was still rather haphazard, which may be related to the poor expression of the two cells themselves. However, we still expected that other scholars would explore this point.

## Figures and Tables

**Figure 1:** The intersection of differentially upregulated genes in keloids but downregulated after hydrocortisone treatment. (a) Differential analysis between keloid samples without hydrocortisone treatment versus normal scar tissue without treatment. (b) Differential analysis between treated and untreated keloid samples. (c) Venn plot of genes not only upregulated in keloid tissue but also downregulated after exposure to hydrocortisone treatment. (d) Major molecular functions of common DEGs enriched based on gene ontology.

**Figure 2:** Expression levels of 22 DEGs in GSE7890 (a) and distinct separation using the expression feature of these 22 DEGs of keloid and nonkeloid lesions in GSE92566: (b) two-dimensional principal component analysis and (c) three-dimensional principal component analysis.

**Figure 3:** Comparison of enrichment scores of fibroblast-related pathways in keloid and nonkeloid lesions contrary to normal scar and their correlations with the expression levels of DEGs.

**Figure 4:** Comparison of immune infiltration scores in keloid and nonkeloid lesions contrary to normal scar and their correlations with individual infiltration scores of immune-related cells. verification of the immune infiltration differences and correlations between key genes and infiltration of immune-related cells in GSE121618.

**Figure 5:** GSEA analyses between keloid lesions and nonlesion keloids based on annotations from hallmark gene sets and c7: immunologic signatures from the molecular signatures database.

**Figure 6:** GSEA analyses between keloid samples expressing high and low levels of *FGF11* (separated by 50% median) based on annotations from hallmark gene sets and c7: immunologic signatures from the molecular signatures database.

**Figure 7:** Expression levels of *IGFBP5* and *FGF11* in different datasets and verification by PCR.

**Table 1:** Functional enrichment analysis (gene ontology) revealed major molecular functions of common DEGs.

Ontology	ID	Description	Gene ratio	*p*	Adjusted *p*	Q
MF	GO: 0005520	Insulin-like growth factor binding	3/18	2.85*e* − 06	2.39*e* − 04	1.74*e* − 04
MF	GO: 0019838	Growth factor binding	3/18	3.40*e* − 04	0.014	0.010
MF	GO: 0044325	Ion channel binding	2/18	0.007	0.098	0.071
MF	GO: 0005178	Integrin binding	2/18	0.008	0.098	0.071
MF	GO: 0019203	Carbohydrate phosphatase activity	1/18	0.010	0.098	0.071

## Data Availability

The datasets generated for this study are available from the corresponding author upon request.
